# Investigation and Analysis of the Key Objectives of WFAS “Technical Specifications of Acupuncture and Moxibustion: General Rules for the Drafting”

**DOI:** 10.1155/2021/9508061

**Published:** 2021-09-22

**Authors:** Zhong-Jie Chen, Jin Huo, Xiao-Yu Wang, Yi Zhang, Jing Hu, Qi Gao, Xiao-Dong Wu, Jing-Jing Wang

**Affiliations:** Institute of Acupuncture and Moxibustion, China Academy of Chinese Medical Sciences, Beijing 100700, China

## Abstract

**Objective:**

To determine the key objectives of WFAS “Technical Specifications of Acupuncture and Moxibustion: General Rules for the Drafting” (hereinafter referred to as General Rules).

**Methods:**

From the medical institutions, colleges, and scientific research organizations at major levels in China and overseas, leading researchers and experts in the field of acupuncture-moxibustion standardization, as well as some experienced foreign specialists in acupuncture-moxibustion, were selected as the respondents. The questionnaire was prepared by using the website of Questionnaire Star, and 60 links of the questionnaire were sent out through e-mail. Excel was used to set up the database and conduct statistical analysis.

**Results:**

Fifty-one valid questionnaires were collected with effective recovery rate of 85%, involving 9 countries (China, South Korea, Italy, Spain, Sweden, Norway, Netherlands, United States, and Canada) from 3 continents. Most experts agreed with us on the target people, structural elements, and text structure proposed in General Rules and held that the General Rules should emphasize the safety and international applicability and should stipulate in details the common problems (contraindications, indications, taboo crowd, target people, therapeutic effects) of various techniques and the specific contents of technical operation (manipulating techniques, selection of patient's body position and treated areas, disinfection and environmental requirements, selection of acupuncture-moxibustion instruments, cautions, needle retention time, treatment frequency, precise location of the acupoints, treatment course) in order to enhance the practicality and operability.

**Conclusion:**

The key objectives of General Rules mainly include target people, structural elements, text structure, safety requirements, common technical problems of acupuncture-moxibustion, and specific details of technical manipulations.

## 1. Introduction

Acupuncture-moxibustion technique has been applied in 183 countries and regions around the world [1]. As a very practical subject, the operational techniques of acupuncture and moxibustion are considered to be extremely important, and the safety and standardization of acupuncture-moxibustion manipulation have always been the major determinants affecting its spread worldwide [2]. Lack of guidance on technical specifications will result in a variety of confusion during operations, leading to a negative impact on the application. At present, there are great variations in the specifications of important acupuncture techniques among countries, such as treatment frequency and the depth of needling. Take acupuncture treatment of osteoarthritis of the knee as an example, some patients are treated once a day or once every other day [3], while other patients being treated once a week [4]. For the protrusion of lumbar vertebra disc, Jiaji acupoints are punctured 50 mm to 75 mm in depth [5], or sometimes shallowly and subcutaneously [6]. Nonuniform and nonstandardized operations will not only affect the effectiveness of acupuncture and moxibustion but also increase the chance of adverse events and even mislead the public understanding and evaluation of acupuncture and moxibustion treatment. Therefore, in order to promote the effective utilization and further development of acupuncture and moxibustion technique in the world, it is very necessary to regulate the technical specifications and formulate international standards in this field.

However, the current international standards for acupuncture and moxibustion technique are quite insufficient. There are only two documents “Standardized Manipulations of Acupuncture and Moxibustion: Part 1 Moxibustion” and “Standardized Manipulations of Acupuncture and Moxibustion: Part 2 Scalp Acupuncture,” published by WFAS in 2012. Few countries have issued national standards or professional standards in this field, including China, Japan, South Korea, the United States, and Australia, with their own focused issues [7]. Except for China, the operation standards in other countries mainly focus on the safety and infection control, while the core technical aspects, such as the procedures and methods of acupuncture and moxibustion related to curative effect, are rarely involved, which is unable to meet the demands of global application of acupuncture technique. Accordingly, it is imperative to formulate international standards for acupuncture and moxibustion technical operation specifications. Compiling the “Technical Specifications of Acupuncture and Moxibustion” to formulate the corresponding international standards is an important measure for the long-term, in-depth, and continuing development of acupuncture-moxibustion [8].

In accordance with international practices, the development of General Rules should be given priority before the formulation of “Technical Specifications of Acupuncture and Moxibustion.” This General Rules is considered to be the basic standard and the basis of other standards within the series. It also offers broad and basic guidance for the formulation of other standards in this series. For this reason, the World Federation of Acupuncture-Moxibustion Societies (WFAS) authorized our research group to host the development of WFAS “Technical Specifications of Acupuncture and Moxibustion: General Rules for the Drafting” (hereinafter referred to as General Rules). Our group has already conducted extensive preliminary survey on the international needs of the General Rules through online questionnaires. In order to reflect the common and key objective problems in the drafting process of “Technical Specifications of Acupuncture and Moxibustion,” to strengthen the guidance and normative effect of the General Rules for meeting the needs of writing specifications of different acupuncture and moxibustion techniques within the worldwide scope, we carried out this investigation. The investigation has further clarified the common goals and issues related to safety and effectiveness in the operation of acupuncture and moxibustion techniques and consulted representative domestic and foreign experts about the related issues. Their opinions will be important basis for forming a new “General Rules” and will provide guidance and reference for the development of specific “standardized manipulations of acupuncture and moxibustion” and lay a foundation for further standardizing acupuncture and moxibustion in clinical operations and promoting a wider application. The results of the survey were analyzed and reported as follows.

## 2. Materials and Methods

### 2.1. Respondents

From the medical institutions, colleges, and scientific research organizations at major levels in China and overseas, leading researchers and experts in the field of acupuncture-moxibustion standardization, as well as some experienced foreign specialists in acupuncture-moxibustion, were enrolled as respondents. It includes seven types of people: leading experts in our research group, the members of WFAS acupuncture standardization working committee, foreign experts from the International Organization for Standardization (ISO)/Chinese Medicine Technical Committee (TC249)/the third and the fourth working groups (WG3 and WG4), the main drafts men of the current criteria of acupuncture and moxibustion, the members of the National Technical Committee on Acupuncture and Moxibustion of SAC, the members of the Third Committee of Standardization Work Committee of Chinese Acupuncture and Moxibustion Society, and acupuncture-moxibustion experts who have been engaged in clinical work abroad for a long time.

### 2.2. Questionnaire Method

The questionnaire was bilingual in Chinese and English. All questions were set as semiopen multichoice ranking questions. The respondents were required to rank each answer according to its importance from highest to lowest on the basis of selecting appropriate answers. Meanwhile, each question was supplemented with a blank option to fill in.

### 2.3. Questionnaire Contents

Our investigation questionnaire concentrated on the key objectives in the developing process of “Technical Specifications of Acupuncture and Moxibustion: General Rules for the Drafting,” aiming at 12 questions, including target people, structural elements, text structure, safety requirements, common problems of acupuncture-moxibustion techniques, specific details of technical manipulations, international applicability, practicality and operability, etc. Different options are listed at the end of each question, and the respondents are required to select the options and rank them according to the importance.

### 2.4. Evaluation of the Reliability and Validity of the Questionnaire

The research group entrusted statistics experts from the Data Center of China Academy of Chinese Medical Sciences to analyze the reliability and validity of this questionnaire.

#### 2.4.1. Reliability Analysis

According to the overall data of the twelve issues in this questionnaire, the research group used SPSS Ver.19.0 to analyze Cronbach's alpha of the questionnaire. The reliability test shows that the alpha coefficient is 0.834 and the alpha coefficient calculated based on standardized data is 0.785, both of the data represent a relatively high level of reliability, indicating that the design of the questionnaire is highly reliable and the results are relatively accurate.

#### 2.4.2. Validity Analysis

The validity is combined by the content validity and face validity. Generally, the KMO value (Kaiser–Meyer–Olkin) and Bartlett's test of sphericity are used to measure the data validity.

Since most of the questions in this questionnaire are multiple choices, the statistical experts believe that the validity analysis is not very suitable for this survey.

Therefore, only some of the questions are involved into the statistical results (such as the third and the eleventh question). All sig values of Bartlett's test of sphericity are 0.000 (<0.05), indicating that the correlation matrix is not an identity matrix. The two parameters of the KMO test statistic are 0.564 and 0.554, which are bigger than 0.5, the recommended standard of the test. Combined with these results, it can be confirmed that the data are suitable for factor analysis and the questionnaire data validity is qualified.

Interpretation of the validity of other issues: all of the issues in this questionnaire are derived from the results of the first-round international demand surveys about the “Technical Specifications of Acupuncture and Moxibustion: General Rules for the Drafting.”

Through the analysis and screening of the survey results, twelve targeted questions (issues) were finally determined. During the formation of this questionnaire, we invited experts who were engaged in the development of relevant standards for acupuncture and moxibustion techniques to participate in the demonstration. After being discussed and optimized by a number of experts in the field, all the items in the questionnaire could express the research content as accurately as possible. The experts assessed that the questionnaire possessed good face validity and content validity.

### 2.5. Investigation Method

This investigation was prepared in both Chinese and English through the platform of electronic questionnaire, the website of Questionnaire Star (https://www.wjx.cn). The questionnaire link was sent through e-mail.

### 2.6. Investigation Time

The preparation and demonstration of the survey questionnaire started from February 9^th^ to 14^th^, 2020. The investigation period is 1 week (February 15～22, 2020) in which two rounds of reply reminders were sent through e-mail, WeChat, and short message service (SMS).From February 22^nd^ to 26^th^, 2020, the original data were exported and statistically analyzed.

### 2.7. Data Sorting and Analysis

Microsoft Excel 14.0 was used to establish a database for statistical analysis.

## 3. Results

### 3.1. Questionnaire Collection

Aimed at the key objectives in General Rules, a total of 60 investigation questionnaires were sent to 11 countries of 4 continents. Among them, 51 valid questionnaire replies were collected from 9 countries of 3 continents, including 2 Asian countries (China 40, South Korea 1), 5 European countries (Italy 2, Spain 2, Sweden 2, Norway 1, the Netherlands 1), and 2 American countries (the United States 1, Canada 1). The collective rate was 85%.

### 3.2. General Information of the Respondents

- Age: averaged 55.69 ± 10.10 years, the youngest 29 years, the oldest 75 years
- Affiliation: 17 people (33.33%) in TCM hospitals, 12 people (23.53%) in medical colleges, 10 people (19.62%) in scientific research institutions, 4 people in TCM clinics and 4 people in specialized hospitals (7.84% respectively), and 2 people in Western medicine comprehensive hospitals and 2 people in private clinics (3.92% respectively)
- Occupation: the majority of participants were Chinese medicine doctors and scientific researchers, including 40 TCM physicians (78.43%), 7 scientific researchers (13.73%), 2 medical teachers (3.92%), and 1 Western medicine physician and 1 in other occupation (1.96% respectively)
- Department: 38 people (74.51%) in acupuncture department, 4 people (7.84%) in TCM department, and 9 people (17.65%) in other departments
- Professional title: 48 people are senior (94.12%), 2 people are intermediate (3.92%), and 1 person is junior (1.96%)
- Working years in the acupuncture-moxibustion field: 30.67 ± 11.18 years on average

### 3.3. The Selection Criteria of the Survey Object (including Identity and Country)

This survey aims at the experts who focus on the research and development of “Technical Specifications of Acupuncture and Moxibustion.” Through preliminary investigations, it is found that only a few foreign experts are specialized in developing the technical standard of acupuncture and moxibustion. Given this situation, the selection criteria are expanded to include domestic experts who focus on developing the technical standard of acupuncture and moxibustion and international experts who are engaged in developing the standards in acupuncture-and-moxibustion-related fields. It is confirmed that authoritative experts in relative fields from all over the world have basically participated in this survey. The participants are as follows:

- Chinese leading researchers who are focused on the technical standard of acupuncture and moxibustion
- Experts in the field of international standards (not limited to the field of acupuncture and moxibustion technical specifications): including SC-WFAS members and foreign representatives of ISO/TC249 WG3 (the group of acupuncture needles) + WG4 (other working groups except for the group of acupuncture needles)
- Foreign experts in the research group
- Foreign experts of acupuncture and moxibustion

Some experts have also been recruited in different organizations, and those duplicate identities have been removed from this survey.

Explanation of the surveyed countries: Considering the different levels of the development of acupuncture and moxibustion in each country, and the uneven distribution of countries participating in the formation of international standard, it turns out that some countries are interested in participating in this survey, while some countries are unwilling to be involved. After excluding those with no response, it can be confirmed that we have already involved sufficient countries and experts that could represent the authoritative group in the field of “Technical Specifications of Acupuncture and Moxibustion” in this survey.

### 3.4. Investigation Results

#### 3.4.1. Target People of General Rules

More than 75% of the experts believed that General Rules should aim at meeting the various needs of the practitioners, compilers, and researchers of the “Technical Specifications of Acupuncture and Moxibustion.”

#### 3.4.2. Structural Elements

More than 70% of the experts believed that General Rules should contain all the structural elements listed in the investigation, as shown in Table 1. The structural elements relating to safety, such as “adverse reactions,” “precautions,” and “contraindications,” occupied the highest proportion of importance, reaching the same level as “cover,” “table of contents,” and “standard title” did (all 94.12%), indicating that experts attached great importance to the safety of acupuncture practice. “Theoretical basis” was in the lowest selection frequency (74.51%). Some experts come up with additional suggestions: (1) editors should be listed and (2) images and videos (electronic version) should be added.

On the basis of the current China's national standard “Technical Specifications of Acupuncture and Moxibustion: General Rules for the Drafting,” it was planned to add two structural elements, “adverse reactions” and “theoretical basis of acupuncture-moxibustion techniques,” and meanwhile, it was stipulated that “diagnosis methods applicable to acupuncture-moxibustion techniques” could be presented in the appendix. With further investigation on these three elements, in order of importance, experts ranked the contents of the “adverse reactions” and “diagnosis methods applicable to acupuncture-moxibustion techniques” and the perspective of demonstration for the “theoretical basis of acupuncture-moxibustion techniques,” as shown in Table 2.

#### 3.4.3. Text Structure

For “from what aspects it should be stipulated in General Rules to ensure the uniformity of the text structure of English version,” the result of investigation is shown in Table 3.

#### 3.4.4. Safety Requirements

Safety is an important requirement that must be contained in all technical specifications [9].

Most experts agreed that, to enhance the safety guiding role of General Rules, the technical specifications of acupuncture and moxibustion should be specified mainly from five aspects, which were ranked from high to low according to experts' opinions, as shown in Table 4.

Some experts put forward that “the overall quality training of acupuncture professionals” and “the definition of the quality of needles” should also be included.

#### 3.4.5. Common Technical Problems and Technical Manipulations to Be Specified in Details

Experts ranked the importance of the common problems covering various acupuncture techniques that need to be detailed in General Rules. The result is shown in Table 5.

For the specific contents of technical manipulations of acupuncture and moxibustion to be detailed, the ranking proposed by experts is shown in Table 6.

#### 3.4.6. Practicability and Operability

Practicability and operability are the important characteristics that all the specifications must stress on. Most experts believed that General Rules should provide detailed descriptions on the practicability and operability of the “Technical Specifications of Acupuncture and Moxibustion” from six aspects, and the ranking from high to low according to experts' opinions is shown in Table 7.

Some experts put forward some additional opinions: (1) “whether the TCM theory could be well understood worldwide” should be considered; (2) to give explanations of origin and development of some acupuncture-moxibustion techniques; and (3) to give descriptions of the qualifications of practitioners using different manipulation methods.

#### 3.4.7. International Applicability

The investigation result of “how to improve the international applicability of General Rules” is shown in Table 8.

## 4. Discussion

According to the result of the first-round investigation of the international demands [10], our research group determined the general scope of the key objective problems to be solved in General Rules and designed the investigation questionnaire accordingly. This investigation effectively collected experts' opinions on the target problems of General Rules and became a key step in the development process of General Rules. The analysis on the investigation result is as follows.

### 4.1. Determine the Target People and Structural Elements and Unify the Text Structure

The result of this investigation clarified that the target people of this General Rules mainly included the global practitioners, compilers, and researchers of the Technical Specifications of Acupuncture and Moxibustion. The expert consensus formed in this survey was that, all the structural elements mentioned in the questionnaire should be included in the Technical Specifications of Acupuncture and Moxibustion; in addition, its text structures should be unified (including “text structure”; “scope and format of terms and definition”; “scope, format, and detailed requirements of the specific content of each part of General Rules”; “expressions of numbers, quantities, units, and values”; “scope and format of bibliography”; “symbols and signs”; “expressions of abbreviated terms”; “linguistic style”).

### 4.2. Attach Great Importance to Safety and Put Forward Specific Requirements

The therapeutic effect and safety of acupuncture and moxibustion are the basis and foundation of its continuous development [11]. Especially for its international application, the safety of acupuncture is the focus of attention [12]. The result of this investigation showed that the structural element “adverse reactions” added in General Rules on the basis of the current China's national standard “Technical Specifications of Acupuncture and Moxibustion: General Rules for the Drafting” (GB/T 33416-2016) has been recognized by most experts. The result of the investigation on the composition of “structural elements” showed that the three structural elements (“adverse reactions,” “precautions,” and “contraindications”) related to safety had the highest degree of expert consensus.

Further investigation into safety revealed that “General Rules” should provide guidance on security of all Technical Specifications of Acupuncture and Moxibustion from five aspects, including “the scope of application of different acupuncture-moxibustion techniques,” “adverse reactions that may occur to different acupuncture-moxibustion techniques,” “contraindications of different acupuncture-moxibustion techniques,” “specification of the operator's qualifications,” and “limitations of acupuncture-moxibustion application by laws and regulations in different countries/regions.” The descriptions of the definition, treatment, prognosis, and causes of “adverse reactions” [13] and other factors can effectively improve the safety control for all technical specifications of acupuncture and moxibustion and avoid the delay of the best time for treatment due to the lack of correct understanding of the safety [14] of acupuncture and moxibustion and adverse reactions. By clearly stipulating the qualifications of practitioners, the clinical disorders caused by unqualified practitioners [15] can be avoided. To ensure the quality of the development of this series of standards, it is essential to emphasize the safety in General Rules, strengthen the security constraints on all the Technical Specifications of Acupuncture and Moxibustion, and promote the safe use of acupuncture and moxibustion in the international scope.

### 4.3. Define the Specific Details of Common Problems and Technical Manipulations of Acupuncture and Moxibustion and Detail the Practicability and Operability

The investigation result showed that most experts agreed to provide the details of the common problems covering multiple acupuncture techniques, including “contraindications,” “indications,” “taboo crowd,” “target patients,” and “therapeutic effects” in General Rules. This can promote the precise application of acupuncture and moxibustion techniques and avoid the side effects caused by improper operation. It coincides with the attention paid by doctors of all dynasties on the “contraindications” of acupuncture and moxibustion [16].

As for the specific content of the technical manipulations of acupuncture and moxibustion, most experts pointed out that all options listed in the investigation should be detailed and explicit, including detailed manipulating techniques (including needle depth and needling sensation), selection of patient's body position and manipulating part, disinfection and environmental requirements, selection of acupuncture-moxibustion instruments, cautions, needle retention time, treatment frequency, precise location of the acupoints, treatment course, etc. In this way, the application of acupuncture and moxibustion techniques can be standardized and restrained more effectively, and the standard manipulation of acupuncture and moxibustion techniques can be guaranteed. At the same time, the specific requirements on the practicability and operability of the Technical Specifications of Acupuncture and Moxibustion should be detailed.

### 4.4. Emphasize the International Applicability

An important role of international standards is to eliminate communication barriers and promote the exchange and development of international technology. Therefore, in the compiling process of the Technical Specifications of Acupuncture and Moxibustion, the General Rules should detail the following contents with full consideration of the differences in the laws and regulations of different countries, requirements of the qualifications of practitioners and their demands, the policy of medical insurance payment systems on acupuncture-moxibustion, the understanding and positioning of acupuncture-moxibustion techniques, preference of acupuncture-moxibustion techniques, and environments. At the same time, it is pointed out that General Rules should stipulate the text of this series of standards from 8 aspects to ensure its unity. All of these will help improve the international applicability of the series of WFAS Technical Specifications of Acupuncture and Moxibustion.

### 4.5. Less Consensus on “Theoretical Basis”

The development and continuous improvement of any kind of technology cannot be separated from the theory guidance. Without the support of theory, technology will lose its foundation. Only by correctly interpreting and inheriting the theory can clinical practice be better guided and improved [17]. Explanation of the “theoretical basis” is helpful for the practitioners to understand the connotation of the applied technology, so as to better grasp its indications and manipulation essentials. It is beneficial to the accumulation and development of the manipulation experience of acupuncture and moxibustion. It is very necessary to add “theoretical basis” for the safe, effective, and standardized use of acupuncture and moxibustion technology. Therefore, the “theoretical basis” was added to the “structural elements” of General Rules. However, the investigation result showed that among all the 18 “structural elements,” the “theoretical basis” was the least frequently selected, indicating that there still existed different viewpoints on whether the “theoretical basis” should be involved in the Technical Specifications of Acupuncture and Moxibustion. This also reflected the current situation of “attaching importance to technology and neglecting theory” in our clinical practice of acupuncture and moxibustion.

### 4.6. Shortcoming of This Investigation

In this investigation, the effective replies of 51 experts from 9 countries (China, Italy, Spain, Sweden, Norway, the Netherlands, the United States, Canada, and Korea)—three continents, Asia, Europe, and the America—were obtained. The sample size was relatively small, and its global representativeness was slightly insufficient. These are the limitations of this investigation. In the follow-up studies, our research group will consult more experts from various countries in order to achieve consensus in a wider range.

## 5. Conclusion

This investigation reveals that the key objectives of General Rules mainly include target people, structural elements, text structure, safety requirements, common technical problems of acupuncture-moxibustion, and specific details of technical manipulations. It provides a valuable reference for the formulation of specific Technical Specifications of Acupuncture and Moxibustion and guarantees the wide application and development of acupuncture and moxibustion technology in the world.

## Figures and Tables

**Table 1:** Investigation of structural elements to be included in General Rules.

Ordering	Options and suggestions	Selection frequency	Percentage (%)
1	Cover	48	94.12
2	Table of contents	48	94.12
3	Title of standards	48	94.12
4	Adverse reactions	48	94.12
5	Cautions	48	94.12
6	Contraindications	48	94.12
7	Terms and definitions	47	92.16
8	Scope	46	90.20
9	Manipulation procedure and rules	46	90.20
10	Manipulating methods	46	90.20
11	Management after manipulation	46	90.20
12	Forward	44	86.27
13	Normative references	44	86.27
14	Preparation before manipulation	44	86.27
15	Introduction	43	84.31
16	Annex	42	82.35
17	Qualifications of manipulators	40	78.43
18	Theoretical basis	38	74.51
19	Other	5	9.80

**Table 2:** Investigation on the contents of three structural elements to be added in General Rules.

Element	Ordering	Options and opinions	Selection frequency	Percentage (%)
“Adverse reactions”	1	Description of adverse reactions	48	94.12
	2	Corresponding measures or recommendations	48	94.12
	3	Definition of the degrees of adverse reactions	44	86.27
	4	Prognosis of adverse reactions	39	76.47
	5	Analysis of the causes of adverse reactions	38	74.51
	6	Other	5	9.80

“Diagnosis methods applicable to acupuncture-moxibustion techniques”	1	Acupoint examination	39	76.47
	2	Special diagnosis methods of special acupuncture-moxibustion methods	38	74.51
	3	Meridian examination	38	74.51
	4	Four diagnostic methods of conventional Chinese medicine	35	68.63
	5	Modern medical diagnostic methods	31	60.78
	6	None of the above choices	6	11.76
	7	Other	2	3.92

“Theoretical basis of acupuncture-moxibustion techniques”	1	From the perspective of traditional Chinese medicine	43	84.31
	2	From the perspective of clinical research	38	74.51
	3	From the perspective of modern medicine	35	68.63
	4	From the perspective of literature	28	54.90
	5	Other	6	11.76

**Table 3:** The English text structure to be stipulated in General Rules.

Ordering	Options and opinions	Selection frequency	Percentage (%)
1	Text structure	49	96.08
2	Scope and format of terms and definition	48	94.12
3	Scope, format, and detailed requirements of the specific content of each part of General Rules	46	90.20
4	Expressions of numbers, quantities, units, and values	44	86.27
5	Scope and format of bibliography	43	84.31
6	Symbols and signs	43	84.31
7	Expressions of abbreviated terms	41	80.39
8	Linguistic style	33	64.71
9	Other	1	1.96

**Table 4:** Investigation of enhancing the safety guiding role of General Rules for the technical specifications of acupuncture and moxibustion.

Ordering	Options and opinions	Selection frequency	Percentage (%)
1	The scope of application of different acupuncture-moxibustion techniques	47	92.16
2	Adverse reactions that may occur to different acupuncture-moxibustion techniques	46	90.20
3	Contraindications of different acupuncture-moxibustion techniques	44	86.27
4	Specification of the operator's qualifications	36	70.59
5	Limitations of acupuncture-moxibustion application by laws and regulations in different countries/regions	32	62.75
6	Other	4	7.84

**Table 5:** Investigation on the common problems covering various acupuncture techniques that need to be detailed in General Rules.

Ordering	Options and opinions	Selection frequency	Percentage (%)
1	Contradictions	47	92.16
2	Indications	44	86.27
3	Taboo crowd	41	80.39
4	Target patients	39	76.47
5	Therapeutic effects	35	68.63
6	Other	2	3.92

**Table 6:** Specific contents of technical manipulations of acupuncture and moxibustion to be detailed in General Rules.

Ordering	Options and opinions	Selection frequency	Percentage (%)
1	Detailed manipulating techniques (including needle depth and needling sensation)	47	92.16
2	Selection of patient's body position and manipulating part	44	86.27
3	Disinfection and environmental requirements	44	86.27
4	Selection of acupuncture-moxibustion instruments	43	84.31
5	Cautions	42	82.35
6	Needle retention time	40	78.43
7	Treatment frequency	40	78.43
8	Precise location of the acupoints	39	76.47
9	Treatment course	39	76.47
10	Other	5	9.80

**Table 7:** Stipulated contents of practicability and operability.

Ordering	Options and opinions	Selection frequency	Percentage (%)
1	Descriptions of various acupuncture-moxibustion techniques' commonness and particularities based on their therapeutic effects	47	92.16
2	The reasons for choosing different acupuncture-moxibustion techniques	44	86.27
3	Manipulations of each technique and it is advisable to give specific examples	40	78.43
4	Key factors of the effectiveness for special acupuncture-moxibustion methods	39	76.47
5	Disinfection requirements of special acupuncture-moxibustion methods	37	72.55
6	Notification of special terms and definitions which are necessary for each part of the technical specification based on the characteristics of individual part	36	70.59
7	Other	6	11.76

**Table 8:** Investigation result of the factors to be considered in improving the international applicability of General Rules.

Ordering	Options and opinions	Selection frequency	Percentage (%)
1	Differences in laws and regulations of different countries	44	86.27
2	Differences in the qualifications of practitioners in different countries	43	84.31
3	Differences in demand of different countries	37	72.55
4	Differences in the policy of medical insurance payment systems in different countries on acupuncture-moxibustion	36	70.59
5	Differences in the understanding and positioning of acupuncture-moxibustion techniques in different countries	35	68.63
6	Differences in acupuncture-moxibustion techniques preferred by different countries	34	66.67
7	Differences in environments of different countries	34	66.67
8	Differences in the definition of tolerance in different countries	28	54.90
9	Other	3	5.88

## Data Availability

The data were taken from the published studies.
